# Microenvironment Stimuli HGF and Hypoxia Differently Affected miR-125b and Ets-1 Function with Opposite Effects on the Invasiveness of Bone Metastatic Cells: A Comparison with Breast Carcinoma Cells

**DOI:** 10.3390/ijms19010258

**Published:** 2018-01-16

**Authors:** Emanuela Matteucci, Paola Maroni, Francesco Nicassio, Francesco Ghini, Paola Bendinelli, Maria Alfonsina Desiderio

**Affiliations:** 1 Dipartimento di Scienze Biomediche per la Salute, Molecular Pathology Laboratory, Università degli Studi di Milano, Milano 20133, Italy; emanuela.matteucci@unimi.it (E.M.); paola.bendinelli@unimi.it (P.B.); 2 Istituto Ortopedico Galeazzi, Scientific Institute for Research, Hospitalization and Health Care (IRCCS), Milano 20161, Italy; paola.maroni@grupposandonato.it; 3 Center for Genomic Science of IIT@SEMM, Istituto Italiano di Tecnologia (IIT), Milano 20139, Italy; francesco.nicassio@iit.it (F.N.); francesco.ghini@iit.it (F.G.)

**Keywords:** Ets-1, HGF, HIF-1α, hypoxia, miR-125b, Endothelin-1, bone metastatic cells

## Abstract

We examined the influence of microenvironment stimuli on molecular events relevant to the biological functions of 1833-bone metastatic clone and the parental MDA-MB231 cells. (i) In both the cell lines, hepatocyte growth factor (HGF) and the osteoblasts’ biological products down regulated nuclear Ets-1-protein level in concomitance with endogenous miR-125b accumulation. In contrast, under hypoxia nuclear Ets-1 was unchanged, notwithstanding the miR-125b increase. (ii) Also, the 1833-cell invasiveness and the expression of Endothelin-1, the target gene of Ets-1/HIF-1, showed opposite patterns under HGF and hypoxia. We clarified the molecular mechanism(s) reproducing the high miR-125b levels with the mimic in 1833 cells. Under hypoxia, the miR-125b mimic maintained a basal level and functional Ets-1 protein, as testified by the elevated cell invasiveness. However, under HGF ectopic miR-125b downregulated Ets-1 protein and cell motility, likely involving an Ets-1-dominant negative form sensible to serum conditions; Ets-1-activity inhibition by HGF implicated HIF-1α accumulation, which drugged Ets-1 in the complex bound to the Endothelin-1 promoter. Altogether, 1833-cell exposure to HGF would decrease Endothelin-1 transactivation and protein expression, with the possible impairment of Endothelin-1-dependent induction of E-cadherin, and the reversion towards an invasive phenotype: this was favoured by Ets-1 overexpression, which inhibited HIF-1α expression and HIF-1 activity. (iii) In MDA-MB231 cells, HGF strongly and rapidly decreased Ets-1, hampering invasiveness and reducing Ets-1-binding to Endothelin-1 promoter; HIF-1α did not form a complex with Ets-1 and Endothelin-1-luciferase activity was unchanged. Overall, depending on the microenvironment conditions and endogenous miR-125b levels, bone-metastatic cells might switch from Ets-1-dependent motility towards colonization/growth, regulated by the balance between Ets-1 and HIF-1.

## 1. Introduction

A complex cross-talk between disseminated breast carcinoma cells and bone marrow niches has been reported [1,2], but the key events for the early metastatic steps and their dependence on the osseous microenvironment are scarcely known. The present paper was designed to evaluate whether stimuli of the bone microenvironment affected the expression of miR-125b and of the target gene Ets-1 [3], influencing the invasiveness and molecular patterns of bone metastatic and parental breast carcinoma cells.

The hepatocyte growth factor (HGF)/Met receptor axis under DNA methylation and miR-34a control plays a critical role in the bone metastatic process of breast carcinoma [4,5]. The pathogenesis of skeleton metastasis implicates an osteoclast–osteoblast interplay mediated by HGF production, responsible for tumour cell migration and seeding into the bone [6]. Osteoblasts represent the major source of HGF, which modulates osteoblastic bone formation and maturation by expressing osteopontin, a non-collagenous component of the extracellular matrix and a cytokine important for proliferation, apoptosis and bone remodelling [6,7]. Supportive cells in vivo release HGF, likely contained in exosomes, affecting bone metastasis outgrowth [4].

Hypoxia and hypoxia inducible factors (HIFs) are important for cancer progression and skeleton metastasis [2,8,9,10], and putative HIF-1 responsive elements (HRE) are present in the promoter of Ets-1, a transcription factor that is the prototype of the ETS family [11]. Several ETS transcription factors are involved in cell malignant transformation and in the progression activating invasion and metastasis-related genes [12]. In human breast carcinoma, Ets-1 enhancement correlates with poor prognosis [13]. In a mouse model, Ets-1 triggers the dissemination of mammary carcinoma cells, regulating the balance between invasion and growth; lung colonization diminishes under Ets-1 overexpression [11].

On the other hand, considering that Ets-1 silencing downregulates Glut1 [13], indirectly affecting the cancer metabolism, and that Ets-1 binding sites are present in the HIF-1α promoter, a relationship between the transcription factors Ets-1 and HIF-1 seems to occur. HIF-1α is the inducible subunit of HIF-1 [9], but other role(s) cannot be excluded.

The novelty of the present paper was to give insight into the regulation exerted by Ets-1 on HIF-1α expression and vice versa, evaluating also the involvement of HIF-1α subunit in Ets-1 transcriptional activity with consequences on the Endothelin-1 signalling in 1833-bone metastatic clone versus parental MDA-MB231 cells, invasive but with low bone tropism [2,8,9,10].

In 1833 cells, HGF downregulates HIF-1 activity at a difference with hypoxia [8,14]. In MDA-MB231 cells, HIF-1 is inactive both under HGF/TGFβ1 and hypoxia because of the downregulation of HIF-1α occurring under HGF/TGFβ1, while hypoxia induces HIF-1α and decreases HIF-1β preventing the active dimer formation [8]. Practically unknown is the role of microenvironment stimuli in the regulation of Endothelin-1 transactivation played by Ets-1/HIF-1 together with other transcription factors, with consensus sequences on Endothelin-1 promoter. 

The signalling pathway orchestrated by Endothelin-1 seems critical for skeleton metastasis formation and prognosis due to E-cadherin augment (adhesion), Runx2 activity and SPARC expression (osteomimicry), occurring only in bone metastatic clone [15,16]. Thus, the Ets-1 control under microenvironment stimuli deserves interest because it might be important for the switch from the invasive phenotype towards osteomimicry and adhesion (both intercellular and to the osteoblastic niche), likely supporting metastatic growth driven by Ets-1/HIF-1-target genes such as Endothelin-1. Various regulators of Ets-1 activity are hypothesized such as growth factors, partner(s) in the DNA binding and miRNAs, since the *ets-1* proto-oncogene does not show rearrangement, amplification or mutation in the primary breast carcinoma [11].

In vitro and in vivo studies show that in breast carcinoma the miR-125 family members are involved in tumorigenesis, playing multiple roles in relation to the intracellular levels: low miR-125b expression correlates with lymph node metastases [3,17]. In the invasive ductal breast carcinoma, the miR-125b promoter shows 48% frequency of methylation, considered as an index of metastatic dissemination [18].

We found that in bone metastatic 1833 clone, but not in MDA-MB231 cells, HGF exposure rapidly increased Ets-1 protein level, returning to the basal value in concomitance with endogenous miR-125b accumulation. Consistently, in HGF-exposed 1833 cells the replenishment of miR-125b with the mimic completely downregulated the Ets-1 protein and invasiveness. The formation of Ets-1-low molecular weight was serum sensible, and might function as a dominant negative [11]. Another molecular regulatory mechanism seemed typical of 1833 cells exposed to HGF: the HIF-1α subunit drugged Ets-1 in the complex bound to Endothelin-1 promoter, preventing Endothelin-1 transactivation; Ets-1 overexpression diminishing the HIF-1α protein level would hamper the negative loop. Altogether, the final result was that the balance between Ets-1 and HIF-1 activities was differently influenced by the microenvironment stimuli, and might affect signals represented by Endothelin-1 and the gene pattern downstream, i.e., E-cadherin enhancement and MMP2 diminution with opposite significance on the invasive phenotype. 

## 2. Results

### 2.1. Different Effects of Stimuli of Bone Metastasis Microenvironment on the Expression of miR-125b, the Ets1 Protein Levels and Invasiveness in MDA-MB231 and 1833 Cells

Here, we addressed the question whether biological characteristics like migration through Matrigel and Endothelin-1 transactivation, were affected by microenvironment stimuli. To clarify the underlying molecular mechanisms, the miR-125b regulatory role towards Ets-1 expression was investigated in 1833-bone metastatic clone and the parental MDA-MB231 breast carcinoma cells exposed to HGF, hypoxia or the conditioned medium of a human osteoblast-like lineage MG-63. The human osteoblasts secrete osteopontin and osteocalcin, that bind cytokines and growth factors, such as HGF, VEGF and TGFβ1 [7,19,20,21,22]. 

As shown in Figure 1A, the MG-63-conditioned medium was added to 1833 and MDA-MB231 cultured cells to evaluate miR-125b expression. The miR-125b basal levels were similar in the two cell lines, and the osteoblast medium increased miR-125b expression more in 1833 than in MDA-MB231 cells. Concomitantly, the Ets-1 protein level decreased of about 60% in both the cell lines, and the following concentrations of growth factors in osteoblast medium were measured: 280 ± 30 pg/mL for HGF, 95 ± 11 pg/mL for TGFβ1 and 110 ± 13 pg/mL for VEGF. 

Next, the experiments were performed in MDA-MB231 cells. Figure 1B reports that the endogenous miR-125b rapidly and transiently doubled under HGF, and under hypoxia strong and persistent enhancements of miR-125b occurred but at later times. The effect of hypoxia on miR-125b expression might be indirect through DNA methyltransferases [23], since MDA-MB231 cells do not show HIF-1 activity [8]. As shown in Figure 1C, HGF caused a fall-down of nuclear Ets-1 protein level at 6–12 h, with a rebound at 18–24 h; hypoxia was ineffective on nuclear Ets-1 protein expression. 

To evaluate the functional significance to the HGF-dependent changes of Ets-1 and the concomitant endogenous miR-125b increase, we studied the effect of miR-125b mimic on MDA-MB231 cell invasiveness. As shown in Figure 1D, the migration through Matrigel decreased under HGF: this effect was enhanced by ectopic miR-125b being inhibitory per se.

Then, the functional study was extended to Endothelin-1 regulation by HGF in MDA-MB231 cells since Endothelin-1 promoter contains 5 Ets-1 and 2 non-canonical HIF-1 binding sites, i.e., HIF-1 and ARNT (Figure 1E). First, we performed the gel-shift with the oligonucleotide for the Ets-1 consensus sequence, and we observed that HGF decreased the Ets-1 DNA binding at 8 h in MDA-MB231 cells. The specific competition with unlabelled probe prevented the binding, while the unspecific competition was ineffective. The super-gel shift experiment with anti-Ets-1 antibody gave immunodepletion of the band, indicating the presence of Ets-1 in the DNA binding complex observed at 4 h. However, the unrelated anti-HIF-1α antibody was ineffective. Second, using the HIF-1 oligonucleotide we observed that the HIF-1-DNA binding was practically absent in MDA-MB231 cells; HGF did not affect the HIF-1 DNA binding, consistent with its inactivity towards HRE multimer (HRELuc) [8]. Using 8-h HGF nuclear extract, the specific competition with unlabelled probe prevented the constitutive binding. Most if not all of the constitutive factor is closely related or identical to the transcription factors ATF-1 and CREB-1 [24,25]. The DNA binding to Octamer-1 oligonucleotide was unaffected by the treatments.

In addition, we observed that in MDA-MB231 cells the HGF treatment persistently downregulated the Ets-1 steady-state protein level (Figure 1F), in agreement with the decreases of Ets-1–DNA binding (Figure 1E) and Ets-1 luciferase activity (Ets1Luc) (Figure 1G upper panel); Ets1Luc was, however, unaffected by HIF-1α expression vector (e.v.) and hypoxia. Figure 1G (lower panel) shows that HGF and hypoxia did not change Endothelin-1 transactivation, and the steady-state protein level of Endothelin-1 remained unchanged under HGF (Supplementary Figure S1).

Further experiments were performed to make a comparison with 1833 cells: nuclear Ets-1 showed two bands of 51 and 52 kDa in MDA-MB231 and 1833 cells [26] (Figure 1F and Figure 2A). In 1833 cells exposed to HGF (Figure 2A), Ets-1 and HIF-1β peaked at 6 h, progressively decreasing until 24 h; HIF-1α biphasically increased at 6 and at 24 h. Differently, hypoxia unaffected Ets-1 protein level, while HIF-1α and β peaked at 6 h (Figure 2A).

Figure 2B shows the pattern of endogenous miR-125b in 1833 cells: a 2-fold increase occurred between 12 and 24 h after HGF, while hypoxia caused an earlier strong and persistent enhancement (3- to 6-fold) from 6 h until 24 h. The graphics report the different effects of the two stimuli (Figure 2C). HGF increased first the Ets-1 protein expression, followed by miR-125b accumulation and Ets-1 fall-down; the endogenous miR-125b expression was elevated under hypoxia but the Ets-1 protein remained at the basal level. Therefore, hypoxia stimulated miR-125b expression unchanging the basal Ets-1-protein levels both in MDA-MB231 and 1833 cells. HIF-1α and β were induced by hypoxia in 1833 cells, while only HIF-1α increased under hypoxia in MDA-MB231 cells [8].

To evaluate whether HGF and hypoxia controlled specific molecular events in bone metastatic cells versus parental breast carcinoma cells, we tested the effects of miR-125b mimic on Ets-1 protein level and cell migration through Matrigel in 1833 cells (Figure 3). Since the two stimuli increased endogenous miR-125b, with the mimic we reproduced this enhancement. 

In a first series of experiments, serum conditions were tested on Ets-1 protein levels in the presence of miR-125b mimic; the tables report the quantitative data and the statistical significance. In total extracts the 27 kDa fragment of Ets-1 was identified, beyond the 51/52 kDa protein [26]. The Ets1 51/52 kDa protein level was higher under 10% FBS than in starved (0.1% FBS) cells and miR-125b reduced it more at 48 h than at 24 h, making the comparison with the respective miR-Control (miR-CTR) and independent of serum conditions. Under starvation, the protein level of the 27 kDa fragment of Ets-1 increased at 24 and 48 h in parallel with the decrease of the precursor protein.

Thus, in 1833 cells the effects of the miR-125b mimic on the Ets-1 forms (precursor or fragment) differed, depending on the serum conditions. 

In next experiments (Figure 3B,C), we examined miR-125b effects on Ets1 protein levels under hypoxia or HGF exposure: the quantitative data and the statistical significance are shown in the histograms. We found that Ets-1 protein levels in hypoxic 1833 cells, transfected with miR-125b mimic, decreased from 24 h until 72 h in respect to hypoxia exposure, becoming similar to the miR-CTR value (Figure 3B). As shown in Figure 3C, 24-h HGF did not modify Ets-1 protein level while ectopic miR-125b, in the presence or the absence of HGF, caused the complete Ets-1 downregulation in 1833 cells.

Altogether, the data of Figure 3A–C suggested that the effect of the miR-125b mimic on Ets-1 protein level depended on the type of stimulus given to bone metastatic cells.

As shown in Figure 3D, after transfection of miR-125b and exposure to 48-h hypoxia, the migration of 1833 cells increased, in respect to hypoxia or ectopic miR-125b alone. Similarly, Ets-1 expression vector (e.v.) stimulated invasiveness, when compared with the control value. 24-h HGF did not modify spontaneous cell migration, which decreased, instead, in the presence of ectopic miR-125b; miR-125b mimic per se was inhibitory on the migration of starved 1833 cells. 

The data confirmed that, under hypoxia and miR-125b, Ets-1 was functional, enhancing the migratory properties of 1833 cells. The diminution of Ets-1 function by miR-125b overexpression under starvation might be due to the 27 kDa fragment working as a dominant negative [11,26]. Of note, HGF diminished Ets-1 protein level in MDA-MB231 but not in 1833 cells.

### 2.2. Reciprocal Regulation of Ets-1 and HIF-1α Transactivating Activities in 1833 Cells

Based on the stimulatory effects of HGF on Ets-1 and HIF-1α protein expression in 1833 cells, we decided to further evaluate Ets-1 activity regulation by the α subunit of HIF-1 and vice versa. In fact, numerous Ets-1 binding sites are present in the HIF-1α promoter, and the Ets1 promoter contains the HIF-1 binding sites HRE (GTGC) and ARNT (CGTC) (Figure 4A). As shown in Figure 4B, the luciferase activity of the HIF-1α-gene reporter without 5’-untranslated region (5′-UTR) was lower than that with the 5′-UTR; Ets1 e.v. reduced the luciferase activity of both the HIF-1α constructs. The 5′-UTR seemed to influence mRNA stability, in agreement with the literature [27]. Figure 4C shows that HGF and the Ets-1 dominant negative (ΔEts1) reduced the activity of HIF-1α promoter with the 5′-UTR: the two treatments showed additive effects. In contrast, HIF-1αLuc activity without the 5′-UTR increased under HGF (Figure 4C), consistent with the enhancement of HIF-1α protein level (Figure 2A); ΔEts1 prevented the luciferase-activity increase indicating a role of the Ets-1 transcription factor in the HGF-dependent enhancement of HIF-1α. ΔEts1 is a partially deleted protein maintaining only the DNA binding domain [28,29]. The transactivating activity of HRELuc was decreased (of about 40%) by Ets-1 e.v. (Figure 4D).

Then, we examined the possible occurrence of an inverse regulation (Figure 4E): Ets-1Luc increased of about 3.5-fold under HGF and doubled after HIF-1α e.v. transfection. Hypoxia was ineffective on Ets-1Luc, consistent with previous data [8].

Notwithstanding the elevated endogenous miR-125b under hypoxia, Ets-1 transactivating activity as well as Ets-1 pro-invasive function were unaffected. Moreover, the increase in the level of the HIF-1α subunit, after expression vector transfection (inset), did not mimic the hypoxic condition because the long-time exposure to hypoxia downregulated, indeed, the HIF-1α and β subunits in 1833 cells. 

### 2.3. Regulation of Endothelin-1 Expression by Microenvironment Stimuli in 1833 Cells

Ets-1 transcription factor might control molecular pathways downstream, such as Endothelin-1 biological signal, through the binding to the consensus sequences present in the promoter. Therefore, we evaluated whether HIF-1α played a role in the Ets-1 binding and whether possible differences occurred between 1833 and MDA-MB231 cells.

As shown in Figure 5A, HGF rapidly accumulated nuclear Ets-1 protein and, therefore, we performed a gel shift assay using proteins extracted early after HGF exposure. The Ets-1 DNA binding to Endothelin-1 promoter was enhanced by HGF at 4 and 8 h; the specific competition with unlabelled probe prevented the binding, while the unspecific competition was ineffective. The super-gel shift with anti-Ets1 and anti-HIF-1α antibodies indicated the presence of these components in the DNA binding complex observed at 4 h (Figure 5B). In contrast, using the HIF-1 oligonucleotide we observed that HGF reduced the HIF-1-DNA binding between 2 and 4 h, with reversion of the effect at 8 h (Figure 5C). The specific competition with unlabelled probe prevented the specific (HIF-1) and constitutive bindings 8 h after HGF. The super-gel shift was performed with anti-HIF-1α antibody, using nuclear extracts from starved and 8-h HGF treated cells; these experiments confirmed the presence of the α subunit in the specific HIF-1 binding complex. Using the ARNT oligonucleotide, we found that HGF diminished principally the constitutive binding at 2 and 4 h; the specific competition prevented the DNA bindings. The super-gel shift with anti-HIF-1α antibody indicated the presence of the α subunit in the HIF-1 specific binding both under starvation and 8-h HGF treatment. The EMSA with HIF-1 and ARNT oligonucleotides showed prominent constitutive bands, impairing a quantitative evaluation.

Taken together, the DNA bindings of Ets-1 and of HIF-1 to Endothelin-1 promoter were oppositely influenced by HGF, in agreement with transactivating activity data of Ets-1Luc and HRELuc (Figure 4E and [14]). The transcription factor regulation and activity seemed to depend on the context of binding sequences involved on the gene promoter [31].

Hypoxia strongly enhanced HIF-1α protein level at 2 and 4 h (Figure 5D); using the HIF-1 and ARNT oligonucleotides, we observed that HIF-1-DNA binding progressively increased from the early times until 8 h of hypoxia exposure (Figure 5E). The super-gel shift with anti-HIF-1α antibody (Ab) confirmed the presence of HIF-1α in the specific bindings under 8-h hypoxia. Specific competition prevented the specific and constitutive bindings. 

The DNA binding to Octamer-1 oligonucleotide was unaffected by the treatments. We did not perform the gel-shift assay of Ets-1 under hypoxic conditions since the Ets-1 protein level and luciferase activity remained unchanged (Figure 2A and Figure 4E).

To further evaluate the molecular regulation of Endothelin-1 expression and function (Figure 6 and Supplementary Figure S2), we studied the transactivating activity of Endothelin-1 under HGF or hypoxia treatment, in respect to basal conditions; since Ets-1 might cooperate with other transcription factors on the promoter, we hindered them with dominant negatives or chemical inhibitors. The effect of Endothelin-1 treatment on the expression of E-cadherin and MMP2 was also examined (Supplementary Figure S2).

As shown in Figure 6A, the basal EndothelinLuc activity was maintained by NF-κB and Fos, as demonstrated by the activity reduction in the presence of SN50, the specific inhibitor of NF-κB [8], or of the c-fos dominant negative (∆Fos). Fos is a subunit of AP-1, and ∆Fos lacks the region encoding amino acid 133 to amino acid 159 of the protein [32]. 

Figure 6B,C report that HGF and hypoxia oppositely affected the luciferase activity of Entothelin650 reporter construct. As shown in Figure 6B, HGF inhibited Endothelin650Luc through HIF-1 and NF-κB activities, since their blockade prevented the inhibitory effect. We co-transfected the EndothelinLuc construct and the dominant negative of the β-subunit (∆Arnt) to inhibit HIF-1 activity and to evaluate its role. In contrast, Ets-1 and Fos dominant negatives gave further inhibition of the Endothelin650Luc activity, probably due to an indirect involvement through a separate signalling pathway. HGF progressively reduced Endothelin-1 protein level until 24 h (inset). Figure 6C shows that hypoxia strongly stimulated Endothelin650Luc: the Ets-1, HIF-1, NF-κB and Fos binding sites in the promoter seemed to be implicated, even if at a different extent. Consistently, hypoxia induced Endothelin-1 protein, peaking at 16 h (inset).

In conclusion, HGF triggered Ets-1 DNA binding while inhibiting HIF-1 DNA binding to Endothelin-1 promoter, and it was ineffective in stimulating Endothelin-1 transactivation and the protein level at the difference with hypoxia (Figure 6D). Altogether, the data indicated the critical importance of the context of binding sequences in the promoter of Endothelin-1 for transcription factor regulation and activity. The inhibition of Ets-1 DNA binding activity was carried out by HIF-1α, and an interplay of HIF-1 and NF-κB seemed to occur in HGF-exposed 1833 cells participating in Endothelin-1Luc activity inhibition.

## 3. Discussion

For the first time we demonstrated that in 1833 bone metastatic cells HGF, a key biological stimulus of microenvironment, remarkably but transiently enhanced the nuclear level of Ets-1, due to the following induction of miR-125b. Differently, in MDA-MB231 cells HGF persistently reduced the nuclear Ets-1 protein level, due to the early miR-125b enhancement, leading to suggest that miR-125b regulation varies with the cell context. There are evidences that the efficacy of miRNAs in degrading mRNA or in decreasing protein synthesis might depend on the complementarity to target mRNAs [17].

In addition, the conditioned medium from an osteoblast-like lineage stimulated miR-125b expression more in 1833 cells than in parental MDA-MB231 cells, reducing Ets-1 protein levels in both the cell lines. Proteomic analysis indicates that osteoblasts secrete molecules for the communication with osteoclasts and for bone remodelling, and that some proteins including growth factors as well as miRNAs are packaged into exosomes [7,19,20,21,22].

Importantly, in 1833 and MDA-MB231 cells under HGF exposure we observed different consequences on biological functions, such as invasiveness and the Endothelin-1 signalling pathway. 

First, HGF inhibited MDA-MB231 cell migration because of the persistent Ets-1 downregulation, while the miR-125b mimic reduced invasiveness of both the cells lines in the absence of serum, notwithstanding HGF addition. The data supported the role of miR-125b in the downregulation of Ets-1 protein level.

Second, HGF exposure enhanced the Ets-1 DNA binding to Endothelin-1 promoter in 1833 cells, but the Endothelin-1 transactivation and the protein levels were unexpectedly reduced. Consistently, only in HGF-treated 1833 cells HIF-1α drugged the Ets-1 in the complex bound to Endothelin-1 promoter. Thus, the Ets-1 transcription factor activity depended on the accumulation of HIF-1α, showing a negative involvement in target-gene expression. HGF enhanced the HIF-1α transactivation (without 5′-UTR) and the protein levels of HIF-1α, which interfered in the Endothelin-1-mediated pro-epithelial function of HGF. Of note, in 1833 cells Endothelin-1 increased E-cadherin expression while reducing MMP2 expression, a pattern similar to that triggered by HGF (Supplementary Figure S2 and Figure 7). Opposite findings were observed in MDA-MB231 cells exposed to HGF, consisting in inhibition of Ets-1 DNA binding to Endothelin-1 promoter, without involvement of HIF-1α.

Based on our data, the adaptability to microenvironment stimuli seemed to be different in bone metastatic versus parental breast carcinoma cells, and the final cell properties under these stimuli might depend on the molecular patterns activated. Methylation state, HIF-1 activity and the responsiveness to HGF differ in parental cells and the bone metastatic clone [4,8]. Now, we show that miR-125b by reducing Ets-1 expression not only affected HIF-1α accumulation and Ets-1 activity, but also HIF-1 activity might be indirectly influenced in HGF-exposed bone metastatic cells.

Hypoxic environment of the bone-marrow (1–7% oxygen) is the preferential site for bone access of metastatic cells disseminated from breast carcinoma [2]. Endogenous miR-125b accumulated in hypoxic 1833 cells, but nuclear-Ets-1 protein level and Ets-1 transactivating activity were unchanged, therefore maintaining the basal values (Figure 7). At support, miR-125b mimic only in part downregulated Ets-1 protein under hypoxia leading to the enhanced Matrigel invasion of 1833 cells. Thus, 1833-cell invasiveness under hypoxia might be explained by miR-125b activity on a partly unknown gene pattern, or directly on transcription factors [17,33]. 

The molecular effects of hypoxia in bone metastatic cells differed from those observed in carcinomas of colon and bladder: in these carcinoma cells, Ets-1 mRNA levels increased under hypoxia, probably due to the decline of expression of Drosha and miRNA biosynthesis [34,35]. 

The bone marrow is hospitable for metastatic cells of breast carcinoma due to staminal, osteoblastic and perivascular niches [1,2,7,16,36], which might be influenced by mild hypoxic conditions and biological stimuli like HGF. Experimental mild hypoxia in 1833 cells causes HIF-1α accumulation with HIF-1 activation [37], without Ets-1 luciferase activity as shown here, suggesting that the co-operation of various transcription factors might play a role in the enhanced expression of target genes, such as Endothelin-1 and E-cadherin (Figure 6, Supplementary Figure S2) [31,38]. As regards Endothelin-1 promoter, the consensus sequences for Fos (AP-1) and NF-κB seemed important for the transactivation under basal conditions and hypoxia, the latter also implicating HIF-1 activity.

Notably, the metastatic cells show a metastable phenotype related also to the interaction between HGF and hypoxia, with a role played by HIF-1α per se (Figure 7). At this purpose, the plasticity of bone metastasis might depend on the activity of transcriptional partners and of miRNAs functioning as co-activators or inhibitors [39]. Various Ets-1 regulatory mechanisms affected the Ets-1 function, which would be important for the switch from invasive to proliferative capacity: HGF mediated the downregulation of Ets-1 transcriptional activity through endogenous miR-125b, HIF-1α accumulation, and the 27 kDa fragment of Ets-1 with dominant negative function in 1833 cells.

Thus, HIF-1α might be considered an Ets-1 interacting protein, to be included in the list of those repressing Ets-1 activity [40]. Also, HIF-1α is an index of poor prognosis of breast carcinoma in human beings [41], independent of HIF-1 transcription factor activity. Notwithstanding the elevated HIF-1α in some cell lines, HIF-1 may be inactive: parental MDA-MB231 cells does not show HIF-1 activity at a difference with the 1833 bone metastatic clone [8]. The regulation of HIF-1α is complex occurring via HDM2, and HIF-1α is also induced by oncogenes [35,42].

Once the migration/engraftment in the bone secondary site has occurred, the metastatic cells assume the epithelial phenotype (MET) important for growth/colonization [43,44,45]: this transcriptional program is likely to be orchestrated by HGF of the microenvironment through Twist phosphorylation [14]. However, HGF-dependent MET phenotype seems to be transient, while being important for metastasis colonization since the proliferation (typical of MET phenotype) prevails on invasiveness [11]. We observed that HGF did not enhance invasiveness of 1833 cells at a difference with hypoxia, and that the basal migration was decreased by ectopic miR-125b also under HGF.

Altogether, the Ets-1 overexpression might facilitate cell motility by preventing HIF-1-dependent Endothelin-1 effects with interference in the E-cadherin mediated adhesive steps of the bone-metastatic process. Ets-1 is known to increase its own transcription and cell invasiveness activating MMPs [34]. A complex interplay of transcription factors seemed to occur under Ets-1 overexpression, which hampered HIF-1α transactivation reducing also HIF-1 activity. Studies are in progress to evaluate the Ets-1 signal in human specimens of breast carcinoma and bone metastasis as well as in the bone-metastasis xenograft model.

## 4. Materials and Methods 

### 4.1. Cell Cultures and miR-125b Transfection

The 1833 bone metastatic clone and the parental invasive MDA-MB231 breast carcinoma cells were kindly given by Dr. J. Massagué (Memorial Sloan-Kettering Cancer Center, New York, NY, USA), and were authenticated with the method of short-tandem repeat profiling (STR) of nine highly polymorphic STR loci plus amelogenin in September 2014 (Cell Service from IRCCS-Azienda Ospedaliera Universitaria San Martino-IST-Istituto Nazionale per la Ricerca sul Cancro, Genova, Italy). The human osteoblast-like cell line MG-63 was purchased from Cell Lines Service (Eppelheim, Germany). All the cells were routinely cultured in DMEM high glucose containing 10% Foetal bovine serum (FBS, Sigma Aldrich, St. Louis, MO, USA) [38,46]. Some 1833 and MDA-MB231 cells were transfected with 30 nM miR-125b (Pre-miR miR-125b Precursor) or miR-CTR (Pre-miR Negative Control 1) [3] (Ambion, Life Technologies, Carlsbad, CA, USA), using Lipofectamine 2000 (Thermo Fisher Scientific, Waltham, MA, USA), according to the manufacturer’s instructions. To prepare the conditioned medium, the MG-63 cells were maintained in culture without serum for 72 h [6]. After the collection, the conditioned medium of four flasks (80 mL) was lyophilized, diluted with starvation medium and added to the flasks with cultured 1833 or MDA-MB231 cells for 24 h. The starvation was performed to avoid the interference of growth factors present in FBS. The ELISA assay (R&D Systems, Abingdon, UK) of HGF, TGFβ1 and VEGF in the conditioned medium was carried out.

### 4.2. Western Blot Analysis

(i) The 1833 and MDA-MB231 cells were starved and treated with 100 ng/mL of HGF (R&D System) [14], or were cultured in 10% FBS and exposed to hypoxia. At various times thereafter, nuclear and total protein extracts were prepared and used for Western blot analysis [30]. (ii) Some cells cultured with 10% FBS were exposed to hypoxia starting 6 h after miR-125b transfection, and were collected at various times thereafter; some starved cells were exposed to HGF for 24 h at the end of the 48-h treatment with miR-125b. Hypoxia (1% oxygen) exposure was performed as reported before [30]. All these cells were used for total protein extracts and Western blot assay. The hybridization of the Western blots was performed with the following antibodies: anti-Ets1 (1:2000, C20, Santa Cruz Biotechnology, Santa Cruz, CA, USA), anti-HIF-1α (clone 54) (1:350, BD-Transduction Laboratories, Franklin Lakes, NJ, USA), anti-HIF-1β (1:200, N19, Santa Cruz Biotechnology), anti-Endothelin-1 (50 ng/mL, Calbiochem^®^ Merck Chemicals Ltd., Nottingham, UK), anti-B23 (1:1000, H106, Santa Cruz Biotechnology), anti-vinculin (1:1000, 4650, Cell Signaling Technology, Beverly, MA, USA). Densitometric analysis was performed after reaction with Enhanced chemiluminescence (ECL) kit from Thermo Fisher Scientific.

### 4.3. Purification of Small RNA Species (miRNAs), and Quantification of miR-125b

Endogenous miR-125b was purified from 1833 and MDA-MB231 cells treated with HGF or hypoxia, or exposed to the conditioned medium from the osteoblastic-like lineage MG-63 cells. miRNAs were isolated through the Maxwell RSC Automated Nucleic Acid Purification System (Promega, Madison, WI, USA) with the Maxwell RSC miRNA tissue Kit (Promega #AS1460). RNA purification of all the samples was checked (260/230 > 2.1; 260/280 > 2.1), and quantified through Nanodrop 2000 (Thermo Fisher Scientific). 1 mg of total RNA was converted to cDNA with the miSCRIPT II RT Kit (Qiagen, Valencia, CA, USA, #216181). RT-qPCR reaction for human miR-125b-5p quantification was performed using 5 ng of cDNA; U6b was used as housekeeping gene. The qPCR run was performed in triplicate, and the data are shown as the means ± S.E. 

### 4.4. Matrigel Invasion Assay

The cells were transfected for 48 h with miR-125b, and were exposed or not to hypoxia or HGF, or were co-transfected with Ets-1 expression vector (e.v.) (1 µg/0.5 mL) (Dr. G. Gambarotta, Dipartimento di Biologia Animale e dell’Uomo, Università degli Studi di Torino, Torino, Italy). HGF was added to the cell cultures for 24 h at the end of the 48-h starvation period in the presence or the absence of miR-125b. For the transfection, the Ets1 e.v. was incubated in a mixture 3:1 of DNA: Fugene 6 (Roche, Basel, Switzerland). The treated cells and the corresponding control cells (cultured for 48 h in the presence of 10% FBS or without serum), were seeded (8 × 10^4^ per well) in the upper chambers of the Matrigel invasion system (BD Biocoat Cellware, Beckton Dickinson Labware, Bedford, MA, USA). The lower chambers contained the culture medium without serum. After 22 h incubation in a humidified tissue culture incubator, non-invading cells were removed from the top, and invading cells were stained with Diff-Quick (Dade Behring, Inc., Newark, NJ, USA). Ten fields were randomly selected for the three replicates, and the number of the cells in each field was counted under 200× magnification [38].

### 4.5. Constructs and Cell Transfections

The cells, seeded in 24-well plates, were transfected with 200 ng/well of the following gene reporters for 24 h: the construct containing the promoter of HIF-1α (−572/+284) with the 5′-UTR and that without the 5′-UTR (−572/+32) (Dr. D.E. Richard, Centre de Recherche, QC, Canada, originally prepared by Dr. G. Semenza, Johns Hopkins University, Baltimore, MD, USA); the construct containing the Endothelin-1 promoter (−650/+173) without the 3′-UTR, prepared in our laboratory from the original construct furnished by Dr. F. Rodriguez-Pascual, Centro Nacional de Investigaciones Biológicas, Madrid, Spain [15]; the multimer construct containing 5 Ets-1 consensus sequences (Ets1Luc) [28], or 6 HRE (HRELuc) (6-HRE, pGL3PGK6TKp), furnished by Dr. P.J. Ratcliffe, Wellcome Trust Centre for Human Genetics, Oxford, UK [14]. As specified, some cells were co-transfected with 1 μg/well of the expression vectors or with 500 ng/well of the dominant negatives: Ets-1 e.v. (Dr. G. Gambarotta); HIF-1α e.v. (Dr. G. Semenza); the dominant negative of Ets-1 (∆Ets1) (∆EBets1, Dr. J. Ghysdael, Institut Curie, Centre Universitaire, Orsey, France); the mutated HIF-1β subunit (∆Arnt, Dr. Schwarz, University of Tübingen, Germany); the ∆Fos (dn-c-fos corresponding to mutated c-fos, Dr. M. Funaba, Kyoto University, Japan) [32]. Some of these transfected cells were concomitantly exposed to hypoxia or to HGF, or were treated with the NF-κB inhibitor SN50 (50 μg/mL, Alexis, Lausanne, Switzerland) [8]. Equivalent amounts of empty vectors were tested. For the transfection of the constructs, we performed an incubation mixture 3:1 of DNA:Fugene 6. In the case of the gene reporters, the mixture contained the internal control pRL-TK (*Renilla* Luciferase Plasmid); Firefly/*Renilla* luciferase activity ratios, calculated by the software, are reported as absolute values [14]. 

### 4.6. EMSA Analysis

Nuclear extracts from cells treated with HGF or exposed to hypoxia were used for gel shift and super-gel shift assays; for the latter, the pre-incubation was performed with 1 μg of anti-Ets1 antibody (15 min at room temperature) or of anti-HIF-1α antibody (OZ12, Thermo Scientific, Freemont, CA, USA) (1 h at 4 °C) [32]. The following labelled oligonucleotides, containing consensus sequences present in the Endothelin-1 promoter, were used: 5′-CTCCGGCTGCACGTTGCCTG-3′, HIF-1 binding site (spanning −414 to −389) [47]; 5′-ACGGCGGGCGTCTGCTTCTG-3′, ARNT binding site (spanning −105 to −86); 5′-AGACATAAAAGGAAAATGAAGCGAG-3′, Ets1 binding site (spanning −414 to −389). The Octamer-1 binding site sequence, used as loading control, was 5′-TGCGAATGCAAAATCACTAGAA-3′. For competition experiments, 50-fold molar excess of each specific double stranded sequence unlabelled, or of an unspecific sequence was added to the binding reaction.

### 4.7. Statistical Analysis

The statistical analysis of the densitometric values for Western blot and EMSA, and of the values for PCR, luciferase activity and cell count of migrated cells, was performed by analysis of variance. The number of independent experiments has been indicated in the legends of the figures. The data are shown as means ± S.E., and their significance was evaluated on the original values in the case of fold variations. *p* < 0.05 was considered significant.

## 5. Conclusions

In the present paper we clarified that the biological and physical stimuli of bone metastasis microenvironment might directly or indirectly regulate transcription factors for metastatic phenotype, also through the involvement of miR-125b, which was an inhibitor of Ets-1 activity and invasiveness under the HGF pro-epithelial stimulus. This molecular mechanism would favour the colonization of metastatic cells homed in bone under the influence of microenvironment signals. 

## Figures and Tables

**Figure 1:** Endogenous miR-125b expression under osteoblast-conditioned medium in 1833 and MDA-MB231 cells, and effects of HGF or hypoxia on miR-125b expression and Ets-1 protein levels and activity in MDA-MB231 cells. (**A**) The conditioned medium from cultured MG-63 osteoblast-like cell line was added to starved 1833 and MDA-MB231 cells (+), and the expression of endogenous miR-125b was evaluated. The relative values were calculated using U6b as housekeeping gene. The experiments have been performed in triplicate, and the means ± S.E. are shown. * *p* < 0.05, ** *p* < 0.005 versus the respective white bar value (untreated cells). (**B**) The expression of endogenous miR-125b was evaluated in MDA-MB231 cells treated with HGF or hypoxia, and the relative values were calculated using U6b as housekeeping gene. The experiments have been performed in triplicate, and the means ± S.E. are shown. * *p* < 0.05 versus starvation value; ** *p* < 0.005, *** *p* < 0.001 versus control value. (**C**) Nuclear protein extracts from MDA-MB231 cells treated with HGF or hypoxia were analysed by Western blot, and immunoreactions were performed with anti-Ets-1 or anti-B23 antibody. The experiments were repeated three times. The densitometric values were normalized with B23, and the data were used to plot the histograms, which show the means ± S.E. of the fold variations versus the first bar, considered as 1. *** *p* < 0.001 versus starvation value. (**D**) Some MDA-MB231 cells were transfected with miR-125b mimic for 48 h, and were exposed or not to HGF for 24 h under starvation. The cells were seeded in the upper chambers, and Matrigel invasion was analysed in the absence of serum. The experiments were performed in triplicate. After cell count in selected fields, the values of migrated cells in 10 fields were calculated, and shown in the graphic as the means ± S.E. for the three replicate. ** *p* < 0.005, *** *p* < 0.001 versus starvation value; ° *p* < 0.05 versus the value in the presence of HGF. (**E**) The consensus sequences for the transcription factors in the Endothelin-1 promoter (−650/+173) are shown. Nuclear extracts, prepared from HGF-treated MDA-MB231 cells, were used for gel-shift assay (EMSA) with the oligonucleotide containing the Ets1 or the HIF-1 consensus sequence. Specific (sp) and unspecific (un) competitions were performed. Super-gel shift was carried out using anti-Ets1 or anti-HIF-1α antibody (Ab), and the nuclear protein extracts from 4-h HGF exposed cells. The experiments were repeated three times. The numbers at the bottom indicate the fold variations versus starvation value, and in the histogram the data are shown as the means ± S.E. * *p* < 0.05 versus starvation value; (**F**) Nuclear protein extracts from MDA-MB231 cells treated with HGF were analysed by Western blot, and immunoreactions were performed with the antibodies shown. B23 was used for normalization. The experiments were repeated three times, and the densitometric evaluation was performed. The numbers at the bottom indicate the fold variations versus starvation value, considered as 1. ** *p* < 0.005, *** *p* < 0.001 versus starvation value; (**G**) The Ets-1 multimer and the Endothelin-1 gene reporter were transfected in MDA-MB231 cells, which were treated as shown. The histograms show the means ± S.E. of experiments performed in triplicate and repeated three times. * *p* < 0.05 versus basal Ets-1 luciferase activity.

**Figure 2:** Effects of HGF and hypoxia on the protein levels of Ets-1 and of the HIF-1 subunits, and on the expression of miR-125b in 1833 cells. (**A**) Nuclear protein extracts from 1833 cells treated with HGF or hypoxia were analysed by Western blot, and immunoreactions were performed with the antibodies shown. B23 was used for normalization. The experiments were repeated three times, and the densitometric evaluation was performed. For each treatment and specific antibody used, the histograms show the means ± S.E. of the relative values, i.e., the fold variations versus the first bar (white) considered as 1. * *p* < 0.05, ** *p* < 0.005, *** *p* < 0.001 versus respective starvation (st) and control (c) values. Red, HGF; blue, hypoxia. (**B**) The expression of endogenous miR-125b was evaluated in 1833 cells treated with HGF or hypoxia, and the relative values were calculated using U6b as housekeeping gene. The experiments have been performed in triplicate, and the means ± S.E. are shown. * *p* < 0.05 versus starvation value; ** *p* < 0.005, *** *p* < 0.001 versus control value; (**C**) We show the time-courses of Ets-1 protein and miR-125b-expression levels: the data are the means ± S.E. * *p* < 0.05, ** *p* < 0.005, *** *p* < 0.001 versus respective starvation and control values. ◊, Ets-1; ■, miR-125b.

**Figure 3:** Effects of ectopic miR-125b on Ets-1 protein levels and invasiveness of 1833 cells. (**A**) Total protein extracts were prepared from 1833 cells exposed to 10% or 0.1% FBS, and transfected with miR-125b mimic or with miR-CTR (control) for 24 or 48 h. Western blot and immunoreactions with anti-Ets1 antibody were performed. Vinculin was used for normalization. The experiments were repeated three times. The Western blots underwent densitometry analysis, and the 51/52 kDa bands were considered together. The tables report the means ± S.E. of the fold variations, and the statistical significance of the data: * *p* < 0.05, ** *p* < 0.005 versus respective control and starvation values. (**B**) Total protein extracts were prepared from 1833 cells transfected with miR-125b mimic or with miR-CTR (control), and exposed to hypoxia for various times starting 6 h after transfection. The experiments were repeated three times, and the histograms show the means ± S.E. of the relative values, i.e., the fold variations versus miR-CTR value. * *p* < 0.05 versus miR-CTR; ^∆^ *p* < 0.05, ^∆∆^ *p* < 0.005 versus respective miR-CTR cells exposed to hypoxia. (**C**) Total protein extracts were prepared from 1833 cells transfected for 48 h with miR-125b mimic or with miR-CTR (control), and exposed to HGF for 24 h. The experiments were repeated three times, and the histogram shows the means ± S.E. of the relative values, i.e., the fold variations versus miR-CTR value: the latter value was similar to that of starvation. *** *p* < 0.001 versus miR-CTR; ^∆∆∆^ *p* < 0.001 versus HGF-exposed cells. (**D**) Some 1833 cells were transfected with miR-125b mimic and were exposed or not to 48-h hypoxia (under 10% FBS) or 24-h HGF (under starvation); other 1833 cells were transfected with Ets-1 expression vector (e.v.). All the cells were seeded in the upper chambers, and Matrigel invasion was assayed in the absence of serum. The experiments were performed in triplicate. After cell count in selected fields, the values of migrated cells in 10 fields were calculated, and shown as the means ± S.E. for the three replicate. * *p* < 0.05 versus hypoxia or HGF value; ^∆^ *p* < 0.05 versus control value. Scale bar = 120 μm.

**Figure 4:** In 1833 cells the transactivation of HIF-1α was affected by Ets-1 e.v. and vice versa. (**A**) The consensus sequences for transcription factors in the HIF-1α and the Ets1 promoters are shown. We used the constructs containing the HIF-1α promoter with or without the 5′-UTR regulatory sequence downstream. After 1833 cell transfection with the HIF-1α promoter constructs, co-transfection was performed (**B**) with the Ets-1 e.v., or (**C**) with the Ets-1 dominant negative (∆Ets1), in the presence or the absence of HGF. We show the means ± S.E. of experiments performed in triplicate, and repeated twice. * *p* < 0.05, ** *p* < 0.005 versus the respective control values of luciferase activity; ° *p* < 0.05 versus HIF-1α (−572/+284) Luc. ^∆^ *p* < 0.05 versus HGF-exposed HIF-1α (−572/+32) Luc. (**D**) The 1833 cells were transfected with the HRE multimer and co-transfected with Ets-1 e.v. We show the means ± S.E. of experiments performed in triplicate, and repeated twice. * *p* < 0.05 versus the control value of HRELuc activity; (**E**) The 1833 cells were transfected with Ets-1 multimer, and co-transfected with HIF-1α e.v. [30], or were exposed to HGF or hypoxia. In the histogram we show the means ± S.E. of experiments performed in triplicate, and repeated twice. * *p* < 0.05 versus the control value of Ets1 activity. Inset: total protein extracts from control (c) and HIF-1α e.v.-transfected cells were used to perform the Western blot, and the immunoblot with anti-HIF-1α antibody. Vinculin was used for normalization. The experiments were repeated three times. The numbers at the bottom indicate the fold variations versus control value. ** *p* < 0.005 versus control value.

**Figure 5:** DNA binding (EMSA) of Ets-1 and HIF-1 under HGF or hypoxia in 1833 cells. (**A**) Nuclear protein extracts, prepared from HGF-treated 1833 cells, were analysed by Western blot and immunoblot with anti-Ets1 antibody was performed. B23 was used for normalization. The experiments were repeated three times. The numbers at the bottom indicate the fold variations versus starvation value, and the histogram shows the data as the means ± S.E. * *p* < 0.05 versus starvation value. (**B**) Nuclear protein extracts, prepared from HGF-treated 1833 cells, were used for gel-shift assay with the oligonucleotide containing the Ets1-consensus sequence. Specific (sp) and unspecific (un) competitions were performed. Super-gel shift was carried out using anti-Ets1 or anti-HIF-1α antibody (Ab), and the nuclear protein extracts from 4-h HGF exposed cells. The experiments were repeated three times. The numbers at the bottom indicate the fold variations versus starvation value, and the histogram shows the data as the means ± S.E. * *p* < 0.05 versus starvation value. (**C**) Nuclear protein extracts, prepared from HGF-treated 1833 cells, were used for gel-shift assay with the oligonucleotides containing the consensus sequence for HIF-1 or ARNT. Specific (sp) competition was performed. Super-gel shift was carried out using anti-HIF-1α antibody (Ab), and the nuclear protein extracts from starved or 8-h HGF exposed cells. The experiments were repeated three times. (**D**) Nuclear protein extracts, prepared from 1833 cells exposed to hypoxia, were analysed by Western blot, and immunoblot with anti-HIF-1α antibody was performed. B23 was used for normalization. The experiments were repeated three times. The numbers at the bottom indicate the fold variations versus control value, and the histogram shows the data as the means ± S.E. *** *p* < 0.001 versus control value. (**E**) Nuclear protein extracts, prepared from 1833 cells exposed to hypoxia, were used for gel-shift assay with the oligonucleotide containing the consensus sequence for HIF-1 or ARNT. Specific (sp) competition was performed; super-gel shift was carried out using anti-HIF-1α antibody (Ab) and the nuclear protein extracts from 8-h hypoxia exposed cells. The experiments were repeated three times.

**Figure 6:** Endothelin-1 transactivation and transcription factor involvement in response to HGF or hypoxia in 1833 cells. (**A**–**C**) The construct containing the Endothelin-1 promoter has been transfected in 1833 cells, which were co-transfected with the dominant negative of Ets1 (∆Ets1), of HIF-1β (∆Arnt) or of Fos (∆Fos), or were exposed to the NF-κB inhibitor SN50, in the presence or the absence of HGF or hypoxia. The histograms show the means ± S.E. of experiments performed in triplicate, and repeated three times. * *p* < 0.05, ** *p* < 0.005, *** *p* < 0.001 versus the respective first bar; ^∆^ *p* < 0.05 versus Endothelin-1Luc exposed to HGF; ^∆∆^ *p* < 0.005, ^∆∆∆^ *p* < 0.001 versus Endothelin-1Luc exposed to hypoxia. Insets: Total protein extracts, prepared from 1833 cells exposed to HGF or hypoxia, were analysed by Western blot and immunoblot with anti-Endothelin-1 antibody was performed [15]. Vinculin was used for normalization. The experiments were repeated three times. The numbers at the bottom indicate the fold variations versus the first lane. * *p* < 0.05 versus starvation or control value. (**D**) Schematic representation of the effects of HGF or hypoxia on the molecular parameters assayed.

**Figure 7:** Involvement of endogenous miR-125b in Ets-1 protein and DNA binding to Endothelin-1 promoter under microenvironment stimuli, and effects on the gene pattern downstream. Pathway activation, +; pathway inhibition, −. In the present paper, the DNA binding and the transactivating activity of Endothelin-1 are used as index of the biological activity of miR-125b on Ets-1 function.

## Supplementary Materials

Supplementary materials can be found at www.mdpi.com/1422-0067/19/1/258/s1.

## Abbreviations

HGF	hepatocyte growth factor
HIF	hypoxia inducible factor
HRE	HIF-1 responsive element
MET	mesenchymal–epithelial transition
